# Smart Medical Prediction for Guidance: A Mechanism Study of Machine Learning

**DOI:** 10.1155/2021/2474473

**Published:** 2021-11-24

**Authors:** Xiangming Wang, Baobao Dong

**Affiliations:** School of Management, Jilin University, Changchun 130025, Jilin, China

## Abstract

Data analysis and prediction have gradually attracted more and more attention in the smart healthcare industry. The smart medical prediction system is of great importance to the enterprise strategy and business development, and it is also of great value to provide medical advices for patients and assist patient guidance. The research theme is the use of machine learning technologies with the application in the areas of smart medical analysis. In this paper, the actual data of the smart medical industry were statistically analysed and visualized according to the features, and the most influential feature combinations were selected for the establishment of the prediction model. Based on machine learning technology, namely, random forest, the guidance prediction model is established, and the combination of features is repeatedly adjusted to improve its accuracy. The practical significance of this paper is to provide a high-precision solution for smart medical data analysis and to realize the proposed data analysis and prediction on the cloud platform based on the Spark environment.

## 1. Introduction

With the development of big data, data analysis and prediction have gradually attracted attention in various industries, and the application of data has become more extensive. Whether in e-commerce, financial transactions, healthcare, or marketing, the use of big data has become a trend. In the era of intelligent medical treatment with the explosive growth of network information, the amount of data to be processed has become larger, the speed of data generation and processing has become faster, the data sources have become more diversified, and the analysis technology of big data has become more complex, flexible, and powerful. This trend has laid a good foundation for the development of smart healthcare.

A cloud platform, also called a cloud computing platform, provides computing, network, and storage capabilities based on hardware and software resources [1]. Cloud computing platforms can be divided into three categories: storage cloud platforms that focus on data storage, computing cloud platforms that focus on data processing, and comprehensive cloud computing platforms that combine computing and data storage processing [2]. Currently, popular cloud platforms include Apache Hadoop and Apache Spark, both of which are distributed computing frameworks based on Hadoop distributed file system (HDFS). Apache Spark is a multilanguage engine for executing data engineering, data science, and machine learning on single-node machines or clusters. Spark can operate at a much faster speed than Hadoop, and its application scope is wider. Therefore, the application of Spark in the smart medical industry has become a wildfire, especially for the analysis and prediction of guidance data [3, 4].

It has become the key to the rapid development of the industry to sort out and summarize the data of the smart medical industry through statistics and analysis and to predict the future trend. With the age approaching, how to live healthily is one of the important issues that modern people pay attention to. Medical guidance data are making healthcare more intelligent through a combination of wireless communication technology, cloud platforms, and the Internet of Things (IoT) and can help patients deal with the problem of improper drug use and medical costs. Through the medical guidance data service, the hospital and doctors can understand the health promotion service status of patients, and the hospital can be promoted from the simple medical function to the role of health promotion. In the era of medical big data, the application of smart medical technology helps to improve medical efficiency and service quality. Through smart medical care, the medical service environment can be improved, and medical resources can be used more properly so that it can give full play to its benefits. In conclusion, medical guidance data can improve the design of information flow, make it easier to manage the medical information system, and provide perfect services for the development of the industry.

According to the above explanation and different needs and goals of patients, doctors, and hospitals, different guidance models are constructed, which also helps smart medical enterprises to make business strategies and business development. Accurate prediction of patient guidance will help smart healthcare companies increase revenue and reduce related costs. In this paper, taking the data of the smart medical industry as an example, the machine learning algorithm is used to analyse and predict the data on the Spark platform, and the accuracy of the prediction is improved to achieve the purpose of the analysis and prediction of the medical guidance data.

## 2. Literature Review

### 2.1. Apache Spark

Apache Spark is an open-source cluster computing framework that was born in 2009 at the University of California, Berkeley, Amplab. Currently, Amplab and Databricks are responsible for the development and maintenance of the entire project, and Spark is being developed by large companies such as Yahoo, Intel, and many other open source enthusiasts. Thousands of companies, including 80% of the Fortune 500, use Apache Spark, over 2,000 contributors to the open-source project from industry and academia. Apache Spark can unify the processing of the data in batches and real-time streaming, using preferred language: Python, SQL, Scala, Java, or R [5]. It can execute fast, distributed ANSI SQL queries for dash-boarding and ad hoc reporting. It runs faster than most data warehouses. It performs exploratory data analysis (EDA) on petabyte-scale data without having to resort to down-sampling and train machine learning algorithms on a laptop and use the same code to scale to fault-tolerant clusters of thousands of machines [6–8].

#### 2.1.1. Spark Core Component

Compared with MapReduce, the first-generation big data ecosystem of Hadoop, Spark has great advantages in terms of performance and consistency of solutions. The Spark framework consists of multiple tightly integrated components. At the bottom is Spark Core which implements Spark's basic functions such as job scheduling, memory management, fault tolerance, and interaction with storage systems. It also provides diversified operations for elastic distributed datasets. Based on Spark Core, Spark provides a series of components for different application requirements, including Spark SQL, Spark Streaming, MLlib, and GraphX. Spark belongs to the subsystem of UC Berkeley's Amplab's BDAS (Berkeley Data Analytics Stack), which aims to build a Hadoop compatible, yet faster and more convenient system. The architecture of the entire BDAS is shown in Figure 1.

As can be seen from Figure 1, Spark SQL is used by Spark to operate structured data. Spark SQL allows users to query data using SQL or Apache Hive SQL dialect (HQL). Spark Streaming is a component of the Spark platform that performs Streaming computing for real-time data and provides rich apis for processing data streams. MLlib is a machine learning algorithm library provided by Spark, which contains a variety of classic and common machine learning algorithms, such as classification, regression, clustering, and collaborative filtering. MLlib not only provides additional capabilities such as model evaluation and data import but also provides some lower-level machine learning primitives, including a general gradient descent optimization algorithm. All of these approaches are designed to scale easily across clusters. GraphX is Spark's graph-oriented computing framework and library. The concept of elastic distributed attribute graph is put forward in GraphX, and on this basis, the organic combination and unification of graph view and table view are realized. Meanwhile, rich operations are provided for graph data processing. Spark focuses on computing data, which is stored in a Hadoop distributed file system called HDFS [9].

In this paper, the machine learning algorithm of Spark MLlib is used to analyse and predict the data. MLlib is a framework for machine learning that provides many types of machine learning algorithms and support model evaluation and data import functions.

#### 2.1.2. RDD

RDD (resilient distributed dataset) is the core element of Spark and abstracts data structure types, and it is the basic computing unit of Spark. It splits data items into collections of partitions, stores them in memory on the working nodes of the cluster, and performs the correct operations. RDD refers to data stored in HDFS, Cassandra, and HBase. Data in other RDD partitions are recalculated in case of a failure or cache recovery. An RDD is a read-only, partitioned collection of records, with each partition distributed on a different node in the cluster. An RDD does not store real data but only a description of data and operations [10, 11].

Figure 2 shows the Spark components interaction flow chart.

As shown in Figure 2, Spark divides the job into stages that are dependent on each other to form a directed acyclic graph (DAG), and a stage contains a series of pipelines.

### 2.2. Machine Learning Algorithms

The objective of this paper is to predict the future guidance situation based on the historical guidance data of smart healthcare. Such application of prediction values is suitable for building prediction models by regression analysis. In this paper, the random forest algorithm is used to establish the prediction model of intelligent medical data.

Ho first proposed random decision forests, which is a classification algorithm containing multiple decision trees. The main concept is to use the sampling process of boostrap to build multiple decision trees and then combine the judgment of multiple decision trees to classify data, so as to avoid the problem of overmatching caused by single decision tree. The generalization characteristic of the whole model is increased to have stronger noise resistance. The random forest machine learning algorithm developed by Leo Breiman and Adele Cutter was a machine learning algorithm consisting of multiple decision trees. An algorithm is based on ensemble learning. The random forest will repeat the sampling every time when the decision tree is established to conduct training in the way of bootstrap [12]. Therefore, each decision tree will receive different training samples. During the training of each decision tree, features will be randomly selected, which is equivalent to feature selection. Based on the above two points, random forest has good versatility and avoids overfitting [7]. As shown in Figure 3, in the regression of random forest, the average of the prediction sum of all decision trees will be calculated and taken as the predicted value of random forest.

## 3. System Architecture and Data Modelling

This paper uses Spark as the main computing framework, YARN as the resource manager, and HDFS as the data storage system. The program is written in Python on PySpark, and the machine learning model is built by using the algorithm of MLlib [11]. The specific steps are shown in Figure 4.

### 3.1. Data Split

First of all, we cut the collected raw data into training data and testing data according to the proportion of 80% and 20%. Training data are the training dataset, which is used to establish the model. Testing data are the test dataset, and the test data are imported into the established model for prediction.

### 3.2. Feature Selection

The selection and processing of features have great influence on the establishment of the training model. Some features of the dataset are useful, while others are useless. Selecting useless features will lead to machine learning bias and less accurate models. Therefore, we use statistical and visual methods to analyse each feature, aiming to find the feature that has the greatest impact on the predicted output, and select the most influential feature combination according to the analysis results for training.

### 3.3. Training Model

Modelling is an iterative process, and we need to carefully look at the combinations of different features, machine learning algorithms, and parameters to find the most appropriate model.

### 3.4. Prediction

The testing data that have been processed are imported into the best model that has been trained for prediction.

### 3.5. Evaluation

In this paper, MAPE (mean absolute percentage error) and RMSPE (root mean square percentage error) were used as evaluation criteria, both of which are common evaluation indexes for the quality of prediction models.

### 3.6. Dataset and Analysis

The dataset used in this article is from the doctor assistant system data of DAOZHENTAI. Doctor sssistant is a new medical decision support system. The goal of the system is to allow doctors to expand the range of differential diagnoses by providing more diagnoses to alert doctors and patients. The physician's assistant can also list the symptoms and tests associated with the clinical condition to help the physician choose a further diagnosis [12]. The medical knowledge base used by physician assistants is established by professional clinicians and adjusted according to actual clinical data.

The data are from 11 hospitals in Zhejiang Province, collected from DAOZHENTAI.COM, from January 1, 2018, to January 1, 2019, for 365 consecutive days, including a total of 37,005 data, and all data are stored as a CSV file. There are eight features, as shown in Table 1.

Date features of the original data are presented in the form of year/month/day, which cannot be directly corresponding to numbers and is not conducive to the establishment of the training model. Therefore, date is extracted into three features, “Year,” “Month,” and “Day,” so as to have a more favourable impact on the training process of machine learning. In this paper, these characteristic values are visualized to facilitate the observation of their trends and to judge the influence of their characteristics on the establishment of the training model.

### 3.7. Modelling

In this paper, the machine learning algorithm of Spark MLlib is used to analyse and predict the data. We analysed and tested the permutations and combinations of different features and finally found the feature with the highest influence for the establishment of the training model [13].

We used the random forest to build the model. Random forest is a highly flexible machine learning algorithm that can be used as a means of dimension reduction to deal with missing values and outliers and assess the importance of features. Random forest establishes a forest in a random way, and the forest is composed of several decision trees. The original data are sampled twice, and different training sets can be obtained in each iteration. Each decision tree will predict the true value, and the tag is the average of the predicted values for the tree [9]. The training model establishment process is as follows:

  randomforestmodel = Random Forest.trainRegressor(traindata,
  categoricalFeaturesInfo = { },
  numTrees = 100,
  featureSubsetStrategy = “auto”,
  impurity = ‘variance',
  maxDepth = 5,
  maxBins = 30)

## 4. Effectiveness Evaluation

### 4.1. Effectiveness Evaluation Methods

In this paper, MAPE and RMSPE were used as performance evaluation criteria. MAPE is the mean absolute percentage error, which is the most common index to evaluate the quality of prediction models. RMSPE is the percentage of root mean square error. MAPE and RMSP are methods to measure the error rate [7–9], so the smaller their scores are, the more accurate the prediction model is. The calculation method is as follows:

(1) MAPE (mean absolute percentage error) is as follows:
  (1) $$\begin{array}{c} \text{MAPE}=\frac{1}{n}\sum_{i=1}^{n}\left|\frac{a_{i}-y_{i}}{a_{i}}\right|. \end{array}$$
(2) RMSPE (root mean square percentage error) is as follows:
  (2) $$\begin{array}{c} \text{RMSPE}=\sqrt{\frac{1}{n}}{\sum_{i=1}^{n}\left(\frac{a_{i}-y_{i}}{a_{i}}\right)}^{2}, \end{array}$$
  where *n* is the total number of days, *a* is the actual value, that is, the receiving income of a hospital in one day, and *y* is the corresponding predicted value.

### 4.2. Results of Effectiveness Evaluation

Firstly, the original data and all the characteristic values (Hospital, Day of week, Date, Sales, Patients, Open, National holiday, School holiday) were used to establish the training model according to the machine learning algorithm. The accuracy of random forest was the highest.

MAPE value of the random forest decreased from 0.31150 to 0.30074, and its error value decreased by 3.5%. The RMSPE value was reduced from 0.50009 to 0.47092, and the error value was reduced by 5.8%. Then, we analysed the influence of each characteristic value on the prediction model and removed the less influential features one by one, such as Open and National holiday. The scores of MAPE and RMSPE in the prediction model were both improved. Finally, we selected Hospital, Day of week, Sales, School holiday, Month, Year, and other features to establish the prediction model, and the MAPE value of random forest decreased from 0.31150 to 0.27398. The error value decreased by 12.0%, RMSPE value decreased from 0.50009 to 0.40755, and error value decreased by 18.5%. See Table 2 for details.

According to the results of MAPE and RMSPE, we found that the data of intelligent medical treatment showed that Hospital, Day of week, Sales, Date, Patients, School holiday, and other factors affected the volume of Hospital referral, which had important significance and value for the analysis and prediction of referral data. In all, the improvement of the index of MAPE and RMSPE can provide more accurate and effective service for doctors and patients. For doctors, they can use the medical guidance data to predict the development of one kind of disease or can know which hospital is good at one aspect. All of these can help hospital and doctors to deal with the right patients and diseases timely and effectively. For patients, they can be saved timely under some urgent conditions, and these medical guidance data can help them find the right doctors and right hospitals to reduce the inappropriate medical treatment, which can improve their health quality.

## 5. Conclusions

Whether it is a set of rules, a tree, or a mathematical equation, machine learning can build models to uncover hidden information in data. Taking the data of the smart medical industry as an example, this paper found that the characteristic values of Hospital, Day of week, Sales, Date, Patients, School holiday, Date, Open, National holiday, and so on all had influences on the status of referral and medical treatment. Among them, Hospital, Day of week, Sales, Date, Patients, and School holiday were the most favourable feature combinations for the establishment of the prediction model.

The prediction model of random forest is highly accurate for predicting the future guidance status of smart medical enterprises. After our experimental improvement, MAPE value is reduced from 0.31150 to 0.27398, and its error value is reduced by 12.0%. RMSPE value decreased from 0.50009 to 0.40755, and the error value decreased by 18.5%. The most important success factors are data preprocessing and feature selection. The original features are improved and extended, and individual most influential feature values are used as training factors of the prediction model.

The mechanism proposed in this paper aims at the continuous data and establishes the prediction model based on the regression analysis method, which is not only applicable to the analysis and prediction of the guidance data in the smart medical industry. In the future, new features can be added to improve the accuracy of the prediction model. For example, weather data have an impact on the number of patients seeking medical treatment and the sales amount of the hospital. In addition, in the face of a larger amount of data, we can use the cloud architecture in this paper to carry out distributed computing. In short, the prediction model of random forest used in this paper is helpful to solve the problem of patient consultation and makes a beneficial exploration for the future consultation model. At the same time, it is also helpful to the strategy implementation and cost reduction of smart medical enterprises. In reality, these data can help doctors set up documents for every patient and each kind of disease. In the near future, smart medical guidance can be improved in some aspects; for example, this way can help patients and doctors identify the right information and deal with these informations effectively, and for the smart healthcare industry, all the medical guidance data can be accumulated to foresee the development directions by enterprises [14].

## Figures and Tables

**Figure 1:** Spark core component architecture.

**Figure 2:** Spark components interaction flow chart.

**Figure 3:** Random forest diagram.

**Figure 4:** System flow chart.

**Table 1:** Data and features.

Features	Value	Type
Hospital	1–11	int64
dayofweek	1–7	int64
Sales	￥0–￥5318	int64
Date	2018/1/1–2019/1/1	object
Patients	0–27339	int64
Open	0, 1	int64
nationalholiday	0, a, b, c	object
schoolholiday	0, 1	int64

**Table 2:** Effectiveness evaluation: MAPE and RMSPE.

	MAPE	Improving rate (%)	RMSPE	Improving rate (%)
Training model	RF		RF	
Raw data	0.31150		0.50009	
Data preprocessing	0.30074	3.5	0.47092	5.8
Remove Open	0.30324	7.4	0.45849	10.2
Remove National holiday	0.27398	9.8	0.40755	13.0

## Data Availability

The data used to support this study are available upon the request.
